The article "DNMT3B decreases extracellular matrix degradation and alleviates intervertebral disc degeneration through TRPA1 methylation to inhibit the COX2/YAP axis" was retracted in 2024. Reasons: results that could not be reproduced; plagiarized images; overlap with other authors' work; signs of a paper mill.

# DNMT3B decreases extracellular matrix degradation and alleviates intervertebral disc degeneration through TRPA1 methylation to inhibit the COX2/YAP axis

**DOI:** 10.18632/aging.203410

**Published:** 2021-08-24

**Authors:** Zhiqiang Luo, Yanchao Ma, Tianning Di, Bing Ma, Hongwei Li, Jiangdong An, Yonggang Wang, Haihong Zhang

**Affiliations:** 1 Department of Orthopedics, Lanzhou University Second Hospital, Lanzhou 730030, P.R. China

**Keywords:** intervertebral disc degeneration, nucleus pulposus, extracellular matrix, inflammation, DNA methyltransferase

## Abstract

Intervertebral disc degeneration (IVDD) is a main cause of low back pain that is associated with extracellular matrix (ECM) degradation and inflammation. This study aims to investigate the role of DNMT3B and its regulatory mechanisms in IVDD. IVDD rat models were constructed followed by transfections with oe-DNMT3B or oe-YAP in order to explore the role of DNMT3B in the development of IVDD. After that transfection, nucleus pulposus (NP) cells were isolated and transfected with oe-DNMT3B, oe-TRPA1, si-YAP, oe-YAP or oe-COX2 in order to investigate the functions of DNMT3B in NP cells. DNMT3B was poorly expressed in IVDD tissues and NP cells whereas TRPA1, COX2, and YAP were highly expressed. The proliferation or apoptosis of NP cells was detected through CCK-8 assay or flow cytometry, respectively. Overexpression of DNMT3B promoted the proliferation of NP cells, inhibited their apoptosis, as well as increasing the expression of collagen II and aggrecan and decreasing expression of MMP3 and MMP9. Besides, DNMT3B suppressed inflammation and alleviated IVDD. Mechanistically, DNMT3B modified the TRPA1 promoter by methylation to inhibit the expression of COX2. Overexpression of COX2 promoted the apoptosis of NP cells and decreased the expression of YAP, which was reversed by upregulating DNMT3B. DNMT3B may promote the proliferation of NP cells and prevent their ECM degradation through the TRPA1/COX2/YAP axis, thereby alleviating IVDD in rats.

## INTRODUCTION

Human intervertebral disc degeneration (IVDD) is a multifactorial process that is caused by both genetic factors and mechanical stress [1]. IVDD is asymptomatic in most cases, and is often correlated with sciatica, spondylolisthesis, disc herniation, and degenerative scoliosis [2]. Currently, clinical interventions for IVDD mainly include conservative medical treatment and surgery, but these treatments only provide temporary relief of painful symptoms [3]. Nucleus pulposus (NP) cells play critical roles in generating aggrecan, type II collagen, and other components of the extracellular matrix (ECM), thereby exerting its important effects on maintaining IVD integrity [4]. During IVDD, pro-inflammatory cytokines such as TNF-α and IL-1β can accelerate NP cell degeneration by promoting the release of matrix metalloproteinases (MMPs) and inflammatory cytokines [5, 6]. Therefore, ECM degradation and inflammation in NP cells have been shown to accelerate the progression of IVDD. However, the underlying factors or mechanisms involved in this process are not yet fully understood.

The article "DNMT3B decreases extracellular matrix degradation and alleviates intervertebral disc degeneration through TRPA1 methylation to inhibit the COX2/YAP axis" was retracted in 2024. Reasons: results that could not be reproduced; plagiarized images; overlap with other authors' work; signs of a paper mill.

DNA methylation is a form of epigenetic modification that plays a crucial role in biological processes. Its multiple functions include; repression of transposons and genes or gene activation, which directly determines disease development [7]. DNA Methyltransferase 3 Beta (DNMT3B) is a major methyltransferase that is known to methylate centromeric, pericentromeric and subtelomeric repeats, while DNMT3B protein plays different roles in diseases that are context-dependent [8]. A recent report indicated that a DNMT3B inhibitor increases the expression of transient receptor potential ankyrin 1 (TRPA1) during erythroid and megakaryocyte differentiation [9]. Additionally, TRPA1 is a cation channel located on the plasma membrane of many types of cells, and is a potential sensor for inflammatory pain [10]. TRPA1 is highly expressed in the intestinal mucosa and exerts anti-inflammatory and protective effects [11]. Moreover, TRPA1 promotes the development of degenerative cartilage changes and joint pain in osteoarthritis, when the expression of a potential mediator, cyclooxygenase 2 (COX-2), gets inhibited [12]. COX-2, a key enzyme in fatty acid metabolism, is induced by pro-inflammatory cytokines and is also a key link in triggering subsequent inflammatory responses [13]. Interestingly, hypoxia increases the expression of COX2 in mesenchymal stem cells, which then activates Yes-associated protein (YAP) in hepatoma carcinoma cells and leads to increased cell proliferation [14]. The dysregulation of YAP is involved in IVDD and cell senescence [15]. Based on the aforementioned evidence, we speculated that DNMT3B might regulate TRPA1/COX2/YAP axis to alleviate IVDD.

## RESULTS

### DNMT3B was lowly expressed in IVDD

Studies have shown decreased DNA methyltransferase DNMT3B expression levels in osteoarthritis [16]. To investigate whether DNMT3B is associated with the development of IVDD, we first constructed a puncture-induced IVDD rat model. H&E and SO staining of the morphology of intervertebral disc tissues revealed decreased numbers of NP cells, chaotic structure of NP cells, and damaged ECM in the IVDD rats relative to that of Sham rats (Figure 1A). Therefore, the histological score of the intervertebral discs of IVDD rats was significantly higher. The levels of collagen II and aggrecan in IVDD rats, indicators of protein degradation of ECM [17], were decreased, while MMP3 and MMP9 levels were increased (Figure 1B, 1C). In addition, IVDD rats exhibited increased levels of inflammatory factors in their intervertebral disc tissues, including IL-6, TNF-α, and IL-8 (Figure 1D). The above results demonstrated that the IVDD rat model was successfully constructed. The mRNA and protein levels of DNMT3B in the IVDD rats were significantly reduced (Figure 1E, 1F), indicating that DNMT3B may be related to the development of IVDD and could probably be a novel biomarker for the condition, which needs to be identified by more comprehensive experiments.

The article "DNMT3B decreases extracellular matrix degradation and alleviates intervertebral disc degeneration through TRPA1 methylation to inhibit the COX2/YAP axis" was retracted in 2024. Reasons: results that could not be reproduced; plagiarized images; overlap with other authors' work; signs of a paper mill.

**Figure 1:** **DNMT3B was expressed in IVDD tissues in low levels.** (**A**) Histological analysis of intervertebral disc tissues of Sham rats and IVDD rats. (**B**) The expression of collagen II, aggrecan, MMP3, and MMP9 detected by RT-qPCR in intervertebral disc tissues of sham-operated rats and IVDD rats. (**C**) Western blot analysis of the expression of collagen II, aggrecan, MMP3, and MMP9 in intervertebral disc tissues of sham-operated rats and IVDD rats. (**D**) The levels of inflammatory factors IL-6, TNF-α, IL-8 was detected by ELISA. (**E**) The expression of DNMT3B in the intervertebral disc of sham-operated rats and IVDD rats was detected by RT-qPCR. (**F**) The expression of DNMT3B in the intervertebral disc of sham-operated rats and IVDD rats was detected by Western blot. Measurement data are expressed as the mean ± standard deviation and analyzed using independent sample t-tests. **, *p* < 0.01.

### Overexpression of DNMT3B promoted NP cell proliferation and reduced ECM degradation and inflammation

To investigate the effects of DNMT3B on NP cells *in vitro*, we isolated and cultured NP cells from the intervertebral disc tissues of IVDD or Sham rats. The NP cells from IVDD or sham-operated rats were paddle-shaped or horn-shaped (Figure 2A). The expression of HIF-1α, HIF-1β, and collagen I in NP cells at passage 1 and 2 from IVDD rats increased with cell passage, while collagen II decreased with cell passage (Figure 2B). These results confirmed that NP cells were successfully isolated from IVDD rats. Moreover, DNMT3B was lowly expressed in NP cells of IVDD rats (Figure 2C, 2D). To study the effects of overexpression of DNMT3B on NP cell proliferation and ECM degradation, NP cells were transfected with oe-DNMT3B, followed by Western blot analysis and RT-qPCR. The results depicted that oe-DNMT3B had significantly increased the mRNA and protein levels of DNMT3B in NP cells (Figure 2E, 2F). More importantly, we found that treatment with oe-DNMT3B had significantly increased the proliferation of NP cells (Figure 2G) but reduced their apoptosis (Figure 2H). Upregulation of DNMT3B expression also reduced the expression of pro-apoptotic factors Bax and caspase-3, but increased that of anti-apoptotic factor Bcl2, which was similar to the control level (Figure 2I, 2J), indicating that the overexpression of DNMT3B enhances the anti-apoptotic ability of NP cells. The balance of ECM synthesis and degradation contributes to the structural stability of the intervertebral disc, which is also a key indicator for evaluating NP cell function [18]. In this assay, we detected the expression of collagen II, aggrecan, MMP3, and MMP9 in NP cells to evaluate the balance of ECM synthesis and degradation of NP cells. As shown in Figure 2K, 2L, oe-DNMT3B increased the expression levels of collagen II and aggrecan, and decreased the expression of MMP3 and MMP9, which was similar to that of the control level. In addition, the results of immunofluorescence staining showed that oe-DNMT3B significantly increased the expression of collagen II (Figure 2M). oe-DNMT3B inhibited inflammation of NP cells as well, as demonstrated by reduced levels of IL-6, TNF-α and IL-8, similar to that of the control level (Figure 2N). Collectively, these results indicated that the overexpression of DNMT3B promoted NP cell proliferation and reduced ECM degradation and inflammation.

The article "DNMT3B decreases extracellular matrix degradation and alleviates intervertebral disc degeneration through TRPA1 methylation to inhibit the COX2/YAP axis" was retracted in 2024. Reasons: results that could not be reproduced; plagiarized images; overlap with other authors' work; signs of a paper mill.

**Figure 2:** **DNMT3B promoted NP cell proliferation and ECM synthesis.** (**A**) Representative images of the morphology of isolated NP cells under an optical microscope. (Scale bar, 100 μm). (**B**) Immunocytochemical staining showing the expression of HIF-1α, HIF-1β, collagen I, collagen II in primary and second generation of NP cells from IVDD rats (scale bar, 50 μm; magnification 200 ×). (**C**) The expression of DNMT3B in NP cells from Sham or IVDD rats was detected by qRT-PCR. (**D**) Western blot showing the expression of DNMT3B in NP cells from Sham or IVDD rats. (**E**) The expression of DNMT3B in NP cells after 24 hours of transfection of oe-DNMT3B was detected by qRT-PCR. (**F**) The expression of DNMT3B in NP cells after 48 hours of transfection of oe-DNMT3B was detected by Western blot. (**G**) The proliferation of NP cells at 24, 48, and 72 hours, after 24 hours of transfection of oe-DNMT3B was detected by CCK-8. (**H**) The apoptosis of NP cells after 48 hours of treatment with oe-DNMT3B was detected by flow cytometry. (**I**) The expression of apoptosis-related factors Bax, Bcl-2, and caspase-3 in NP cells after 24 hours of treatment with oe-DNMT3B was detected by qRT-PCR. (**J**) The expression of apoptosis-related factors Bax, Bcl-2, and caspase-3 in NP cells after 48 h ours of transfection with oe-DNMT3B was detected by Western blot. (**K**) The expression of collagen II, aggrecan, MMP3, and MMP9 in NP cells after 24 hours of transfection with oe-DNMT3B was detected by RT-qPCR. (**L**) The expression of collagen II, aggrecan, MMP3, and MMP9 in NP cells after 48 hours of transfection with oe-DNMT3B was detected by Western blot. (**M**) Immunofluorescence staining showing the protein content of collagen II in NP cells after 48 hours of treatment with oe-DNMT3B. (**N**) The levels of inflammatory factors IL-6, TNF-α, IL-8 in NP cells after 24 hours of treatment with oe-DNMT3B were detected by ELISA. Measurement data are expressed as the mean ± standard deviation (n = 3) and analyzed using independent sample t-tests between two groups or using two-way ANOVA between groups at different time points. **, *p* < 0.01.

The article "DNMT3B decreases extracellular matrix degradation and alleviates intervertebral disc degeneration through TRPA1 methylation to inhibit the COX2/YAP axis" was retracted in 2024. Reasons: results that could not be reproduced; plagiarized images; overlap with other authors' work; signs of a paper mill.

### DNMT3B inhibited the expression of TRPA1 by modifying TRPA1 promoter methylation

A study has shown that DNMT3B inhibits the expression of TRPA1 during erythroid and megakaryocyte differentiation [9]. TRPA1 is highly expressed in the intervertebral disc after being treated with pro-inflammatory cytokines, and may participate in the homeostasis of the intervertebral disc [19]. To verify whether DNMT3B works in a TRPA1-dependent manner, we first used RT-qPCR and Western blot to detect the expression of TRPA1 in the intervertebral disc tissues of IVDD rats. As shown in Figure 3A, 3B, the mRNA and protein levels of TRPA1 in the IVDD rats were significantly increased. Functional experiments were conducted to further identify the role of TRPA1, by transfecting NP cells with oe-NC or oe-DNMT3B. As shown in Figure 3C, 3D, oe-DNMT3B reduced the mRNA and protein levels of TRPA1, indicating that DNMT3B might inhibit the expression of TRPA1. Next, C-phosphate-G (CpG) island was identified in the TRPA1 promoter region through the UCSC Genome Browser Database website (http://genome.ucsc.edu) (Figure 3E). The addition of aza (a DNMT3B inhibitor) reduced the methylation of the TRPA1 promoter (Figure 3F), and the overexpression of DNMT3B could promote the methylation of the TRPA1 promoter. In addition, aza reversed the promotion of DNMT3B on the methylation of the TRPA1 promoter. As shown in Figure 3G, aza increased the luciferase reporter gene activity of the TRPA1-WT promoter, while oe-DNMT3B reduced the luciferase reporter gene activity of the TRPA1-WT promoter. Fascinatingly, aza reversed the inhibition of DNMT3B on the luciferase reporter gene activity of the TRPA1-WT promoter. However, at the same time, there was no significant change in the luciferase reporter gene activity of the TRPA1-MUT promoter (Figure 3G). The application of aza resulted in the decreased expression of DNMT3B and an increase in the expression of TRPA1, while oe-DNMT3B had the opposite effects. aza reversed the inhibition of oe-DNMT3B on the expression of TRPA1 (Figure 3H, 3I). These data indicated that DNMT3B inhibited the expression of TRPA1 by promoting the methylation of TRPA1 promoter.

The article "DNMT3B decreases extracellular matrix degradation and alleviates intervertebral disc degeneration through TRPA1 methylation to inhibit the COX2/YAP axis" was retracted in 2024. Reasons: results that could not be reproduced; plagiarized images; overlap with other authors' work; signs of a paper mill.

**Figure 3:** **DNMT3B inhibited the expression of TRPA1 through methylation.** (**A**) RT-qPCR showing the expression of TRPA1 in the intervertebral disc tissue of IVDD rats (n = 10) and sham-operated rats (n = 10). (**B**) Western blot showing the expression of TRPA1 in the intervertebral disc tissue of IVDD rats). (**C**) mRNA expression of DNMT3B and TRPA1 in NP cells after 24 hours of transfection with oe-DNMT3B or oe-NC was detected by RT-qPCR. (**D**) mRNA expression of DNMT3B and TRPA1 in NP cells after 48 hours of transfection with oe-DNMT3B or oe-NC was detected by Western blot. (**E**) A C-phosphate-G (CpG) island in the TRPA1 promoter region was identified in UCSC website. (**F**) The methylation of the TRPA1 promoter was measured through MSP in NP cells after 24 hours of transfection with oe-DNMT3B. (**G**) The luciferase reporter assay of luciferase activity in promoter of the TRPA1-WT and TRPA1-MUT in NP cells after 24 hours of transfection with oe-DNMT3B. (**H**) RT-qPCR showing the mRNA expression of DNMT3B and TRPA1 in NP cells after 24 hours of transfection with aza or oe-DNMT3B. (**I**) Western blot showing the protein expression of DNMT3B and TRPA1 in NP cells after 48 h treatment with aza or oe-DNMT3B. Measurement data are expressed as the mean ± standard deviation (n = 3) and analyzed using independent sample t-tests between two groups or using one-way ANOVA between multiple groups. **, *p* < 0.01; ns, not significant.

### DNMT3B inhibited TRPA1 to promote NP cell proliferation and to reduce its ECM degradation and inflammation

To explore the effect of DNMT3B on NP cells by inhibiting the expression of TRPA1, we transfected NP cells with oe-NC, oe-TRPA1, or oe-DNMT3B. As shown in Figure 4A, 4B, oe-DNMT3B reversed the promotion of oe-TRPA1 on mRNA and protein levels of TRPA1, while the overexpression of TRPA1 hardly altered the expression of DNMT3B. Additionally, oe-TRPA1 reduced the proliferation of NP cells and increased their apoptosis, and additional treatment of oe-DNMT3B had the opposite effects (Figure 4C, 4D). Increased TRPA1 levels elevated the expression of pro-apoptotic factors Bax and caspase-3 and reduced the expression of anti-apoptotic factor Bcl2, and further treatment of oe-DNMT3B reversed these changes (Figure 4E, 4F). Moreover, results from RT-qPCR and immunofluorescence revealed that oe-TRPA1 reduced the expression of collagen II and aggrecan but increased the expression of MMP3 and MMP9; however, the addition of oe-DNMT3B restored the expression of MMP3, MMP9, collagen II and aggrecan (Figure 4G–4I). These alterations supported the inhibitory effect of DNMT3B on ECM degradation through the inhibition of TRPA1. Furthermore, oe-TRPA1 increased the expression of IL-6, TNF-α, and IL-8, but addition of oe-DNMT3B reversed the effects (Figure 4J). These data indicated that DNMT3B promoted the proliferation of NP cells and reduced their ECM degradation and inflammation in a TRPA1-dependent manner.

The article "DNMT3B decreases extracellular matrix degradation and alleviates intervertebral disc degeneration through TRPA1 methylation to inhibit the COX2/YAP axis" was retracted in 2024. Reasons: results that could not be reproduced; plagiarized images; overlap with other authors' work; signs of a paper mill.

**Figure 4:** **DNMT3B inhibited TRPA1 to regulate NP cell proliferation and ECM degradation.** (**A**) The expression of DNMT3B and TRPA1 in NP cells after 24 hours of treatment with oe-DNMT3B or oe-TRPA1 was detected by RT-qPCR. (**B**) The expression of DNMT3B and TRPA1 in NP cells after 48 hours of treatment with oe-DNMT3B or oe-TRPA1 was detected by Western blot. (**C**) The proliferation of NP cells after 24 hours of treatment with oe-DNMT3B or oe-TRPA1 was detected by CCK-8. (**D**) The apoptosis of NP cells after 48 hours of treatment with oe-DNMT3B or oe-TRPA1 was detected by flow cytometry. (**E**) The expression of apoptosis-related factors Bax, Bcl-2, and caspase-3 was detected by qRT-PCR in NP cells after 48 hours of treatment with oe-DNMT3B or oe-TRPA1. (**F**) The expression of apoptosis-related factors Bax, Bcl-2, and caspase-3 was detected by Western blot in NP cells after 48 hours of treatment with oe-DNMT3B or oe-TRPA1. (**G**) The expression of collagen II, aggrecan, MMP3, and MMP9 was detected by RT-qPCR in NP cells after 48 hours of treatment with oe-DNMT3B or oe-TRPA1. (**H**) The expression of collagen II, aggrecan, MMP3, and MMP9 was detected by Western blot in NP cells after 48 hours of treatment with oe-DNMT3B or oe-TRPA1. (**I**) Immunofluorescence staining showing collagen II protein in NP cells after 48 hours of treatment with oe-DNMT3B or oe-TRPA1. (**J**) Inflammatory factors IL-6, TNF-α, IL-8 levels in NP cells after 24 hours of treatment with oe-DNMT3B or oe-TRPA1 were detected by ELISA. Measurement data are expressed as the mean ± standard deviation (n = 3) and analyzed using one-way ANOVA between multiple groups or using two-way ANOVA between groups at different time points. **, *p* < 0.01; ns, not significant.

### DNMT3B regulated the proliferation, apoptosis and ECM degradation of NP cells via TRPA1-COX2 axis

Studies have shown that the activation of TRAP1 promotes the expression of COX2 in osteoarthritis [12], and that COX2 is highly expressed in inflammatory cytokine-mediated IVDD [20]. Thus, we detected the expression of COX2 in the intervertebral disc tissues of Sham rats or IVDD rats. The mRNA and protein levels of COX2 in the IVDD rats were significantly increased, as shown in Figure 5A, 5B. To investigate whether DNMT3B inhibits the expression of COX2 through TRPA1, we transfected NP cells with oe-TRPA1 or oe-DNMT3B. As shown in Figure 5C, 5D, oe-TRPA1 increased the mRNA and protein levels of TRPA1 and COX2, which was reversed by additional treatment with oe-DNMT3B, indicating that DNMT3B can inhibit the expression of COX2 through TRPA1.

The article "DNMT3B decreases extracellular matrix degradation and alleviates intervertebral disc degeneration through TRPA1 methylation to inhibit the COX2/YAP axis" was retracted in 2024. Reasons: results that could not be reproduced; plagiarized images; overlap with other authors' work; signs of a paper mill.

**Figure 5:** **DNMT3B regulated NP cell proliferation and ECM degradation by inhibiting TRPA1-COX2 axis.** (**A**) The expression of COX2 in the intervertebral disc tissue of IVDD and Sham rats was detected by RT-qPCR (n = 10). (**B**) Western blot showing the expression of COX2 in the intervertebral disc tissue of IVDD and Sham rats. (**C**) mRNA expression of DNMT3B, TRPA1, and COX2 in NP cells after 24 hours of treatment with oe-DNMT3B and oe-TRPA1 was detected by qRT-PCR. (**D**) Protein expression of DNMT3B, TRPA1, and COX2 in NP cells after 48 hours of treatment with oe-DNMT3B, oe-TRPA1 or oe-NC was detected by Western blot. (**E**) DNMT3B, TRPA1, and COX2 mRNA expression in NP cells after 24 hours of treatment with oe-DNMT3B, oe-COX2 or oe-NC detected by RT-qPCR. (**F**) DNMT3B, TRPA1, and COX2 protein expression in NP cells after 48 hours of treatment with oe-DNMT3B, oe-COX2 or oe-NC detected by Western blot. (**G**) The proliferation of NP cells after 24 hours of treatment with oe-DNMT3B, oe-COX2 or oe-NC was detected by CCK-8 assay. (**H**) The apoptosis of NP cells after 48 hours of treatment with oe-DNMT3B or oe-COX2 was detected by flow cytometry. (**I**) The expression of apoptosis-related factors Bax, Bcl-2, and caspase-3 was detected by qRT-PCR in NP cells after 24 hours of treatment with oe-DNMT3B or oe-COX2. (**J**) The expression of apoptosis-related factors Bax, Bcl-2, and caspase-3 was detected by Western blot in NP cells after 48 hours of treatment with oe-DNMT3B or oe-COX2. (**K**) The expression of collagen II, aggrecan, MMP3, and MMP9 was detected by qRT-PCR in NP cells after 24 hours of treatment with oe-DNMT3B or oe-COX2. (**L**) The expression of collagen II, aggrecan, MMP3, and MMP9 was detected by Western blot in NP cells after 48 hours of treatment with oe-DNMT3B or oe-COX2. (**M**) Immunofluorescence staining showing collagen II protein in NP cells after 48 hours of treatment with oe-DNMT3B or oe-COX2. (**N**) Inflammatory factors IL-6, TNF-α, IL-8 levels in NP cells after 24 hours of treatment with oe-DNMT3B or oe-COX2 were detected by ELISA. Measurement data are expressed as the mean ± standard deviation (n = 3) and analyzed using independent sample t-tests between two groups, using one-way ANOVA between multiple groups, or using two-way ANOVA between groups at different time points. **, *p* < 0.01.

The article "DNMT3B decreases extracellular matrix degradation and alleviates intervertebral disc degeneration through TRPA1 methylation to inhibit the COX2/YAP axis" was retracted in 2024. Reasons: results that could not be reproduced; plagiarized images; overlap with other authors' work; signs of a paper mill.

To explore the effect of DNMT3B on NP cell proliferation and ECM degradation through the TRPA1/COX2 axis, NP cells were transfected with oe-COX2 or oe-DNMT3B. As shown in Figure 5E, 5F, oe-DNMT3B can reverse the promotion of oe-COX2 on mRNA and protein levels of COX2. Additionally, oe-COX2 reduced the proliferation of NP cells and increased their apoptosis, which can be impaired by oe-DNMT3B (Figure 5G, 5H). Increased COX2 was found to induce the expression of pro-apoptotic factors Bax and caspase-3 and reduced the expression of anti-apoptotic factor Bcl2, and further treatment of oe-DNMT3B reversed those changes (Figure 5I, 5J). oe-COX2 reduced the expression of collagen II and aggrecan but increased the expression of MMP3 and MMP9, and further treatment of oe-DNMT3B had the opposite effects (Figure 5K, 5L), which was consistent with the results of immunofluorescence staining of collagen II (Figure 5M). Furthermore, the expression of IL-6, TNF-α, and IL-8 can be enhanced by oe-COX2 and reduced by oe-COX2 + oe-DNMT3B (Figure 5N). The aforementioned results suggested that DNMT3B promoted the proliferation of NP cells and reduced the cells’ ECM degradation and inflammation properties in a COX2-dependent manner.

### COX2-mediated YAP affects NP cell viability and ECM degradation

Studies have shown that COX2 overexpression promotes the expression of YAP [21], which is highly expressed in IVDD [15]. In this study, we first detected the expression of YAP and found that the mRNA and protein levels of YAP in the IVDD rats were significantly increased (Figure 6A, 6B).

**Figure 6:** **COX2 promoted YAP/Hippo signaling pathway to promote NP cell proliferation.** (**A**) The expression of YAP in the intervertebral disc tissue of IVDD and sham-operated rats was detected by RT-qPCR (n = 10). (**B**) Western blot showing the expression of YAP in the intervertebral disc tissue of IVDD and sham-operated rats. (**C**) The interference efficiency of si-YAP in NP cells after 24 hours of transfection was detected by RT-qPCR. (**D**) The interference efficiency of si-YAP in NP cells after 48 hours of transfection was detected by Western blot. (**E**) mRNA expression of COX2 and YAP in NP cells after 24 hours of transfection with oe-COX2 and si-YAP was detected by RT-qPCR. (**F**) COX2 and YAP protein expression in NP cells after 48 hours of transfection with oe-COX2 and si-YAP was detected by Western blot. (**G**) The proliferation of NP cells after 24 hours of transfection with oe-COX2 or si-YAP was detected by CCK-8. (**H**) The apoptosis of NP cells after 48 hours of transfection with oe-COX2 or si-YAP was detected by flow cytometry. (**I**) The expression of apoptosis-related factors Bax, Bcl-2, and caspase-3 was detected by RT-qPCR in NP cells after 24 hours of transfection with oe-COX2 or si-YAP. (**J**) The expression of apoptosis-related factors Bax, Bcl-2, and caspase-3 was detected by Western blot in NP cells after 48 hours of transfection with oe-COX2 or si-YAP. (**K**) The expression of collagen II, aggrecan, MMP3, and MMP9 was detected by qRT-PCR in NP cells after 24 hours of transfection with oe-COX2 or si-YAP. (**L**) The expression of collagen II, aggrecan, MMP3, and MMP9 was detected by Western blot in NP cells after 48 hours of transfection with oe-COX2 or si-YAP. (**M**) Immunofluorescence staining showing collagen II protein in NP cells after 48 hours of transfection with oe-COX2 or si-YAP. (**N**) Inflammatory factors IL-6, TNF-α, IL-8 levels in NP cells after 48 hours of transfection with oe-COX2 or si-YAP were detected by ELISA. Measurement data are expressed as the mean ± standard deviation (n = 3) and analyzed using independent sample t-tests between two groups, using one-way ANOVA between multiple groups, or using two-way ANOVA between groups at different time points. **, *p* < 0.01.

The article "DNMT3B decreases extracellular matrix degradation and alleviates intervertebral disc degeneration through TRPA1 methylation to inhibit the COX2/YAP axis" was retracted in 2024. Reasons: results that could not be reproduced; plagiarized images; overlap with other authors' work; signs of a paper mill.

To study the effect of COX2-mediated YAP protein in the Hippo signaling pathway on NP cell proliferation and ECM degradation, NP cells were transfected with oe-NC + si-NC, oe-COX2 + si-NC, oe-NC + si-YAP, or oe-COX2 + si-YAP. Firstly, we designed three si-YAP sequences. The expression of YAP after treatment of si-YAP-3 was the lowest, so the si-YAP-3 sequence was selected for subsequent experiments, as shown in Figure 6C, 6D. According to Figure 6E, 6F, si-YAP reduced the expression of YAP, and oe-COX2 reversed the effect of si-YAP. si-YAP increased the proliferation of NP cells and reduced their apoptosis, which could be impaired by oe-COX2 (Figure 6G, 6H). si-YAP reduced the expression of pro-apoptotic factors Bax and caspase-3 and increased the expression of anti-apoptotic factor Bcl2, and further treatment of oe-COX2 exhibited opposite effects (Figure 6I, 6J). Moreover, si-YAP rescued the reduced expression of collagen II and aggrecan and yet increased the expression of MMP3 and MMP9 by oe-COX2 (Figure 6K–6M), as demonstrated by RT-qPCR and immunofluorescence. si-YAP reduced the expression of IL-6, TNF-α, and IL-8, and further treatment of oe-COX2 had the opposite effects (Figure 6N). These findings supported that COX2 suppressed the proliferation of NP cells and enhanced their ECM degradation and inflammation properties in a YAP-dependent manner.

The article "DNMT3B decreases extracellular matrix degradation and alleviates intervertebral disc degeneration through TRPA1 methylation to inhibit the COX2/YAP axis" was retracted in 2024. Reasons: results that could not be reproduced; plagiarized images; overlap with other authors' work; signs of a paper mill.

### DNMT3B affected NP cell viability and ECM degradation via COX2-mediated YAP

In order to explore whether DNMT3B regulated the Hippo signaling pathway through COX2, NP cells were transfected with oe-NC, oe-COX2, or oe-DNMT3B.

According to Figure 7A, 7B, oe-COX2 increased the expression of COX2 and YAP, and further treatment of oe-DNMT3B had the opposite effects, indicating that DNMT3B can regulate the expression of YAP through COX2.

**Figure 7:** **DNMT3B promoted NP cell proliferation and ECM synthesis via COX2-YAP axis.** (**A**) DNMT3B, TRPA1, COX2, and YAP expression in NP cells after 48 hours of treatment with oe-DNMT3B and oe-COX2 was detected by RT-qPCR. (**B**) DNMT3B, TRPA1, COX2, and YAP expression in NP cells after 48 hours of treatment with oe-DNMT3B and oe-COX2 was detected by Western blot. (**C**) DNMT3B, TRPA1, COX2, and YAP expression in NP cells after 48 hours of treatment with oe-DNMT3B and oe-YAP was detected by RT-qPCR. (**D**) DNMT3B, TRPA1, COX2, and YAP expression in NP cells after 48 hours of treatment with oe-DNMT3B and oe-YAP was detected by Western blot. (**E**) The proliferation of NP cells after 48 hours of treatment with oe-DNMT3B or oe-YAP was detected by CCK-8. (**F**) The apoptosis of NP cells after 48 hours treatment with oe-DNMT3B or oe-YAP was detected by flow cytometry. (**G**) The expression of apoptosis-related factors Bax, Bcl-2, and caspase-3 was detected by RT-qPCR in NP cells after 48 hours of treatment with oe-DNMT3B or oe-YAP. (**H**) The expression of apoptosis-related factors Bax, Bcl-2, and caspase-3 was detected by Western blot in NP cells after 48 hours of treatment with oe-DNMT3B or oe-YAP. (**I**) The expression of collagen II, aggrecan, MMP3, and MMP9 was detected by RT-qPCR in NP cells after 48 hours of treatment with oe-DNMT3B or oe-YAP. (**J**) The expression of collagen II, aggrecan, MMP3, and MMP9 was detected by Western blot in NP cells after 48 hours of treatment with oe-DNMT3B or oe-YAP. (**K**) Immunofluorescence staining showing collagen II protein in NP cells after 48 hours of treatment with oe-DNMT3B or oe-YAP. (**L**) Inflammatory factors IL-6, TNF-α, IL-8 levels in NP cells after 48 hours of treatment with oe-DNMT3B or oe-YAP were detected by ELISA. Measurement data are expressed as the mean ± standard deviation (n = 3) and analyzed using one-way ANOVA between multiple groups or using two-way ANOVA between groups at different time points. **, *p* < 0.01.

The effects of DNMT3B-COX2-YAP axis on NP cell proliferation and ECM degradation were identified by transfecting NP cells with oe-NC, oe-YAP, or oe-DNMT3B, followed by experiments including CCK-8, flow cytometry, RT-qPCR and Western blot analysis to assess capacities of apoptosis, proliferation and ECM. As shown in Figure 7C, 7D, oe-YAP increased the expression of YAP, and oe-DNMT3B could reverse the effect of oe-YAP. Additionally, oe-YAP reduced the proliferation of NP cells and increased their apoptosis, which could be enhanced by oe-DNMT3B (Figure 7E, 7F). oe-YAP increased the expression of pro-apoptotic factors Bax and caspase-3 and reduced the expression of anti-apoptotic factor Bcl2, and further treatment of oe-DNMT3B restored the expression of Bax, Bcl2 and caspase-3 (Figure 7G, 7H). Moreover, oe-YAP reduced the expression of collagen II and aggrecan, but increased the expression of MMP3 and MMP9, and further treatment of oe-DNMT3B had the opposite effects (Figure 7I, 7J), which was consistent with the results of the immunofluorescence staining of collagen II (Figure 7K). oe-YAP increased the expression of IL-6, TNF-α, and IL-8, which can be rescued by oe-DNMT3B (Figure 7L). The results demonstrated that DNMT3B promoted the proliferation of NP cells and enhanced their ECM synthesis through the COX2-YAP axis.

The article "DNMT3B decreases extracellular matrix degradation and alleviates intervertebral disc degeneration through TRPA1 methylation to inhibit the COX2/YAP axis" was retracted in 2024. Reasons: results that could not be reproduced; plagiarized images; overlap with other authors' work; signs of a paper mill.

### DNMT3B alleviated IVDD through TRPA1/COX2/YAP axis

To study the roles of the TRPA1-COX2-YAP axis in DNMT3B alleviating IVDD in rat models, IVDD rats were injected with NP cells with oe-NC, oe-YAP, or oe-DNMT3B. As shown in Figure 8A, 8B, oe-DNMT3B increased the expression of DNMT3B, and reduced the expression of TRPA1/COX2/YAP, and oe-YAP can rescue the effect of oe-DNMT3B on YAP. H&E and SO staining were used to stain the intervertebral disc tissues of each group of rats. According to Figure 8C, the number of NP cells in rats injected with NP cells with oe-YAP was reduced and the NP structure became disordered, while oe-DNMT3B could rescue the effects of oe-YAP. The results of SO staining showed that oe-DNMT3B could reverse the destructive effects of oe-YAP on ECM. The treatment with oe-YAP increased the histological score of intervertebral disc (Figure 8C), whereas oe-DNMT3B reduced the score, indicating that contrary to oe-YAP, oe-DNMT3B alleviated the symptoms of IVDD. Moreover, oe-YAP reduced the expression of collagen II and aggrecan, and increased the expression of MMP3 and MMP9, and further treatment of oe-DNMT3B had the opposite effects (Figure 8D, 8E). oe-YAP increased the expression of IL-6, TNF-α, and IL-8, and further treatment of oe-DNMT3B could impair the expression of IL-6, TNF-α, and IL-8 (Figure 8F). The results indicated that DNMT3B prevented the development of IVDD through TRPA1-COX2-YAP axis.

**Figure 8:** **DNMT3B alleviated IVDD through TRPA1-COX2-YAP axis.** Seven days after IVDD surgery, rats were injected with oe-DNMT3B and/or oe-YAP lentivirus vectors by tail vein for 3 consecutive days. Rats were euthanized 4 weeks after IVDD surgery, and C4-C6 intervertebral disc tissues were collected. (**A**) DNMT3B, TRPA1, COX2, and YAP expression in IVDD rats treated with oe-DNMT3B and oe-YAP was detected by RT-qPCR. (**B**) DNMT3B, TRPA1, COX2, and YAP expression in IVDD rats treated with oe-DNMT3B and oe-YAP were detected by Western blot. (**C**) Histological analysis of the intervertebral disc tissue. (**D**) The expression of collagen II, aggrecan, MMP3, and MMP9 was detected by RT-qPCR in intervertebral disc tissues of rat models treated with oe-DNMT3B or oe-YAP. (**E**) The expression of collagen II, aggrecan, MMP3, and MMP9 was detected by Western blot in intervertebral disc tissues of rat models treated with oe-DNMT3B or oe-YAP. (**F**) Inflammatory factors IL-6, TNF-α, IL-8 levels were detected by ELISA in intervertebral disc tissues of rat models treated with oe-DNMT3B or oe-YAP. Measurement data are expressed as the mean ± standard deviation (n = 3) and analyzed using one-way ANOVA between multiple groups. **, *p* < 0.01.

The article "DNMT3B decreases extracellular matrix degradation and alleviates intervertebral disc degeneration through TRPA1 methylation to inhibit the COX2/YAP axis" was retracted in 2024. Reasons: results that could not be reproduced; plagiarized images; overlap with other authors' work; signs of a paper mill.

## DISCUSSION

IVDD, the main cause of low back pain that may lead to disability, is increasingly becoming the focus of medical attention [22]. Although IVDD is mainly attributed to the decrease in the number of NP cells, current treatment strategies (surgery and conservative treatments) still cannot increase the number NP cells or reverse the pathology [23]. Therefore, it is imperative to explore the molecular mechanism underlying IVDD. In this study, we clarified that inducing the expression of DNMT3B increased proliferation and reduced apoptosis of NP cells, ECM degradation, and inflammation. Mechanistically, DNMT3B methylated TRPA1, and TRPA1/COX2/YAP mediated the protective effect of DNMT3B on NP cells. In IVDD rat models, we further confirmed that the overexpression of DNMT3B could alleviate the number and structure of NP cells. Hence, our findings indicated that DNMT3B/TRPA1/COX2/YAP may be a new therapeutic target for IVDD (Figure 9).

**Figure 9:** **Diagram illustrating the pathway of our proposed hypothetical mechanism.** DNMT3B reduces the levels of MMP3 and MMP9 and increases the levels of collagen II and aggrecan through the TRPA1-COX2-YAP axis. DNMT3B then reduces the ECM degradation of NP cells and the inflammatory response, thereby alleviating IVDD.

Because vasculature atrophies with age, the intervertebral disc itself is susceptible to degeneration [24]. The imbalance between ECM metabolism and inflammatory response in NP tissues is a key culprit in the development of IVDD [25]. The ECM of NP tissues is rich in collagen and proteoglycans [26]: Type II collagen and aggregated proteoglycans, and are involved in water uptake, nutrient diffusion, and osmoregulation in NP tissues [27]. A coordinated balance between the catabolic and anabolic aspects of the ECM gradient is essential to proper structure and function of the intervertebral disc [28]. In IVDD, imbalanced ECM metabolism presents as the loss of type II collagen and proteoglycans, altered morphology and structure of intervertebral disc, reduced water content and mechanical buffering capacity [29, 30]. Aging and degeneration lead to multiple biological changes in intervertebral disc cells, including altered cell type in the NP, elevated cell density but reduced amount of living cells [31]. More importantly, it has been demonstrated that intradiscal injection of CHOP shRNA inhibits apoptosis of intervertebral disc cells and suppresses disc degeneration [32]. In the present study, we explored the mechanisms behind these cellular phenotypic changes. It has been shown that DNMT3B enhances inflammation in alcohol-induced liver injury via TRAF2 [33]. We found that the mRNA and protein levels of DNMT3B were significantly reduced in the intervertebral disc tissues of the IVDD rats. Furthermore, we performed gain-of-function and loss-of-function tests on DNMT3B and confirmed that DNMT3B could promote the proliferation of NP cells and inhibit ECM degradation, thus decreasing expression of inflammatory cytokines TNF-α, IL-6 and IL-8 and content of MMP3 and MMP93. Pro-inflammatory cytokines play an important role in the development of IVDD by promoting ECM degradation. IL-1β and TNF-α not only act directly as injurious triggers, but also activate the expression of other potentially injurious molecules, including IL-6 and IL-8 [34]. IL-6 activates the signal transducer and activator of transcription 3 in NP cells to induce IVDD by increasing the expression of MMP [35, 36]. It seems that silencing IL-1β, TNF-α, IL-6 and IL-8, accompanied with decreased expression of MMP, could hinder the progression of IVDD, which supports the inhibitory effect of DNMT3B on the disease development.

The article "DNMT3B decreases extracellular matrix degradation and alleviates intervertebral disc degeneration through TRPA1 methylation to inhibit the COX2/YAP axis" was retracted in 2024. Reasons: results that could not be reproduced; plagiarized images; overlap with other authors' work; signs of a paper mill.

It is well known that DNMT3B adds a methyl group at the cytosine portion of DNA to regulate gene expression [37]. Inhibition of TRPA1 expression is attenuated by DNMT3B inhibitor during erythroid and megakaryocyte differentiation [9], in which TRPA1 is involved in the regulation of the inflammatory response and ECM homeostasis in intervertebral disc [19]. Elderly mice have IVDD whose L4/L5 lumbar dorsal root ganglia exhibit an accumulation of TRPA1 channels [38]. In this study, we found enhanced methylation levels of the TRPA1 promoter upon overexpression of DNMT3B, by luciferase reporter assay. In line with previous research [19], our functional experiments indicated that TRPA1 promoted apoptosis, ECM degradation, and inflammation of NP cells. TRPA1 is known to be a non-selective cation channel, and is expressed in sensory nerves, keratinocytes, mast cells, dendritic cells, and endothelial cells where TRPA1 also acts as a receptor for injury and enhances inflammation [39]. For example, mRNA expression levels of interleukins such as IL-6 were reduced in TRPA1^KO^ mice, suggesting that TRPA1 is a major contributor to the inflammatory process [40]. TRPA1 receptor also enhances intracellular Ca2^+^ concentration to promote apoptosis in oligodendrocytes [41].

As far as inflammatory responses are mediated by TRPA1, many reports have referred to the role of COX-2. TRPA1 agonists inhibit COX-2 in lung cancer cells and suppress hypoxia-induced inflammation [42]. TRPA1 mediates the anti-inflammatory effects of N-Acylethanolamine in a COX-2-dependent manner in rheumatoid arthritis [43], as inactivation of COX-2 and other mediators is associated with alleviation of IVDD [44]. In addition, through gain-of-COX2 and/or TRPA1 function, the evidence of the current study indicated that COX2 promoted apoptosis of NP cells and upregulated IL-6, TNF-α, IL-8 as well as the expression of Bax and caspase-3, which was reversed by overexpression of DNMT3B. It has been shown that YAP suppresses COX2 to induce cellular remodeling of pulmonary artery smooth muscle cells [45]. YAP1 is a member of the Hippo pathway, regulating various cellular processes, such as cell proliferation, contact inhibition, and tissue size [46, 47]. YAP1 overexpression induced degeneration and upregulated the Col-II and aggrecan expression while YAP1 inhibitor effectively impeded the development of IVDD. IL-6 enhanced the interaction of YAP1 and β-catenin and nuclear accumulation [48]. We also noted that silencing YAP1 decreased the content of inflammatory factors and ECM-related factors in NP cells and IVDD rats, but the overexpression of COX2 reversed these alterations, findings that are consistent with previous studies.

In conclusion, this study demonstrated that DNMT3B impeded the development of IVDD through TRPA1/COX2/YAP1 axis. We believe that the newly discovered DNMT3B/TRPA1/COX2/YAP1 axis may provide more insight into the understanding of the potential molecular mechanisms and provide an attractive target for new therapies of IVDD.

## MATERIALS AND METHODS

### Ethical statement

All animal experiments were performed with the approval of the Animal Ethics Committee of Lanzhou University Second Hospital. The experiments involving animals were conducted in accordance to the recommendations in the Guide for the Care and Use of Laboratory Animals of the National Institutes of Health. All experiments were approved by the ethics committee of Lanzhou University Second Hospital.

The article "DNMT3B decreases extracellular matrix degradation and alleviates intervertebral disc degeneration through TRPA1 methylation to inhibit the COX2/YAP axis" was retracted in 2024. Reasons: results that could not be reproduced; plagiarized images; overlap with other authors' work; signs of a paper mill.

### IVDD rat model construction

A total of 60 adult male Speaque Dawley (SD) rats (aged two months and weighing 200-250 grams), purchased from Experimental Animal Center of Lanzhou University Second Hospital [authorization number: SCXKI (Hu) 2017-0005; Lanzhou, China], were raised under a specific pathogen-free environment at 22–24° C with 50–60% humidity and a 12 hour light/dark cycle. After 2 weeks of adaptation, fifty rats were selected to construct IVDD models [49]. Briefly, rats were anesthetized using 2% (w/v) pentobarbital sodium (40 mg/kg, Sigma-Aldrich, CA, USA), and midline incisions were made in the rats’ posterior cervical vertebrae by incising skin and subcutaneous tissues. The paravertebral muscles were exposed and each layer of muscle was completely isolated. The supraspinous and interspinous ligaments of rat cervical alignment (C2-C7) were removed, followed by the suturing of subcutaneous fascia and skin in a specific way to allow suture lines to fall off naturally. The other ten rats were subjected to sham surgery (sham-operated rats) only with the incision of the posterior cervical spine and closure. All rats were monitored during recovery. Rats were intraperitoneally injected with penicillin at 80,000 U/day after three days of surgery. After 4 weeks, rats were euthanized with excess 4% pentobarbital sodium, and C4-C6 of rats was collected under a microscope for subsequent experiments.

### Lentivirus injection in IVDD rat models

The lentiviral transfection complex was diluted according to the instructions of the transfection reagent (En-transterTM-*in vivo*). Seven days after IVDD surgery, 40 rats were injected with 3 μL of phosphate buffer saline (PBS) containing 0.5 nM lentivirus loaded with overexpressed DNMT3B (oe-DNMT3B) + oe-negative control (NC), oe-NC + oe-YAP, oe-DNMT3B + oe-YAP, and oe-NC respectively (n = 10) for 3 consecutive days, while 10 rats were injected with the same volume of control lentiviruses. All plasmids were synthesized by Shanghai Genechem Co., Ltd., (Shanghai, China). Four weeks after IVDD surgery, the rats were euthanized with excess 4% pentobarbital sodium, and C4-C6 of IVDD was collected under the guidance of a microscope for subsequent experiments.

### Isolation, culture, and identification of rat NP cells

The NP tissues were isolated from the rats’ intervertebral disc tissues, washed and cut into pieces under sterile conditions. The NP tissues were left to digest with 0.25% trypsin at 37° C for 10 minutes, centrifuged for 5 minutes, treated with 0.2% collagenase II and centrifuged again for 5 minutes. After the separation of NP cells, they were cultured in Dulbecco's modified eagle medium (DMEM)/F12 medium containing 10% FBS (Gibco), 100 ug/ml streptomycin, and 100 U/ml penicillin in an incubator at 37° C and 5% CO_2_. The medium was changed every three days. The NP cells were collected and sub-cultured in a culture dish after reaching 80–90% confluence, and the NP cells at passage 2 were used for subsequent assays. The expression of HIF-1α, HIF-1β, collagen I and collagen II in NP cells was identified by immunocytochemistry. The cells were fixed in 4% formaldehyde, treated with 0.5% Triton X-100 for 15 minutes, and incubated with 3% H_2_O_2_ for 15 minutes at room temperature. Cells were then left to block in 5% goat serum at 37° C for 30 minutes, and incubated with rabbit anti-HIF-1α (ab51608, 1:2000, Abcam, Cambridge, UK), mouse anti-HIF-1β (ab2771, 1:500, Abcam, Cambridge, UK), mouse anti-type I collagen (ab90395, 1:1000, Abcam, Cambridge, UK), and mouse anti-type II collagen (ab185430, 1:1000, Abcam, Cambridge, UK) at 4° C overnight. Afterwards, the cells were incubated with goat anti-rabbit and goat anti-mouse secondary antibodies labeled with biotin for 30 minutes at room temperature, developed with diaminobenzidine, and counterstained with hematoxylin. Subsequently, the cells were sealed with neutral gel and observed under a microscope.

The article "DNMT3B decreases extracellular matrix degradation and alleviates intervertebral disc degeneration through TRPA1 methylation to inhibit the COX2/YAP axis" was retracted in 2024. Reasons: results that could not be reproduced; plagiarized images; overlap with other authors' work; signs of a paper mill.

### NP cell transfection

One day before transfection, NP cells in the logarithmic growth phase were seeded into a six-well plate with a density of 4×10^5^ cells/well. NP cells were transfected with oe-DNMT3B, oe-TRPA1, si-YAP (si-YAP-1, si-YAP-2, si-YAP-3), oe-YAP, oe-COX2 and the corresponding negative controls (oe-NC, si-NC) using lipofectamine 2000 (11668-019, Invitrogen, NY, CA, USA) after reaching approximately 80%-90% confluence. The aforementioned plasmids, vector construction, sequencing identification, and virus packaging were constructed by Shanghai Genechem Co., Ltd., (Shanghai, China). NP cells were collected for subsequent studies after being incubated for 48 hours.

### Histological analysis

Four weeks after the operation, rats were euthanized by the intraperitoneal injection of 4% pentobarbital, and the rats’ C4-C6 tissue samples were subsequently harvested. The samples were later were decalcified, fixed in formaldehyde, dehydrated, embedded in paraffin, cut into 5 um slices, and stained with Safranin O (SO) and Hematoxylin and Eosin (H&E). The morphology of the tissues was double-blindly examined under a microscope (Olympus Corporation, Tokyo, Japan) by other experienced histology researchers and was evaluated using a grading scale. Histological scores of normal intervertebral disc, moderately degenerated disc and severely degenerated disc were 5, 6–11, and 12–14 [50], respectively.

The article "DNMT3B decreases extracellular matrix degradation and alleviates intervertebral disc degeneration through TRPA1 methylation to inhibit the COX2/YAP axis" was retracted in 2024. Reasons: results that could not be reproduced; plagiarized images; overlap with other authors' work; signs of a paper mill.

### Cell counting kit-8 (CCK-8) assay

Pre-heated 150 μl α-MEM medium containing 10% CCK-8 solution (96992, Sigma, USA) was added to 96-well plates, with a well as the blank control being added with only a mixture of α-MEM and CCK-8. The plate was incubated at 37° C for 2 hours for detecting the optical density (OD) value (at 450 nm) after 24 hours, 48 hours, and 72 hours. The experiment was repeated three times and the average value was calculated.

### Flow cytometry

Forty-eight hours after transfection, the cells were digested with 0.25% trypsin (without EDTA) (YB15050057, YBio Co., Ltd., Shanghai, China). The Annexin-V-FITC, PI, and HEPES buffer solutions were mixed into Annexin-V-FITC/PI staining solution at a ratio of 1:2:50 according to the instructions of Annexin-V-FITC Apoptosis Detection Kit (K201-100, Biovision, CA, USA). Cells were resuspended in staining solution at 1×10^6^/100 μL, incubated at room temperature for 15 minutes, and added with 1 mL of HEPES buffer solution (PB180325, Procell, Wuhan, China). The FITC and PI fluorescence were detected for the evaluation of cell apoptosis and ModFit LT software (Verity software House) was used for analysis. FITC and PI fluorescence was detected by 525 and 620 nm band-pass filters at a wavelength of 488 nm.

### Enzyme-linked immunosorbent assay (ELISA)

After the tissues and cells were lysed by cell lysate, the homogenous supernatant of intervertebral disc tissues was collected following centrifugation and the cell culture supernatant was subsequently collected. The protein concentration was measured using the BioRad Bradford protein assay kit. The ELISA kit (WuHan AmyJet Scientific Inc., Wuhan, Hubei, China) was used for the determination of interleukin-6 (IL-6, No. K4143-100) and tumor necrosis factor alpha (TNF-α) (No. K1051-100), IL-8 (No. K4169-100) in intervertebral disc tissues and NP cells. According to the instructions, the sample was packaged, fixed, blocked, and subjected to protein binding and streptomycin treatment. OD value was measured at the wavelength of 450 nm with a microplate reader. The sample concentration was calculated by drawing a standard curve.

### Immunofluorescence staining

The NP cells were washed twice with PBS, left to fix with 3.5% formaldehyde at 37° C for 30 minutes, permeabilized with 0.1% Triton X-100 in PBS for 20 minutes, and blocked with 3% bovine serum albumin (BSA) and 0.05% Tween 20 in PBS for 30 minutes at room temperature. After cells were left to block, they were incubated at 4° C overnight with rabbit polyclonal anti-collagen II (4 μg/mL, ab34712, 1:1000, Abcam, Cambridge, UK), and incubated with goat anti-rabbit secondary antibodies (2 μg/mL, ab150077, 1:1000, Abcam, Cambridge, UK) for 1 hour at room temperature. The nuclei were stained with 4’,6-diamidino-2-phenylindole (DAPI) and the samples were visualized by a confocal laser scanning microscope (Leica, Wetzlar, Germany).

The article "DNMT3B decreases extracellular matrix degradation and alleviates intervertebral disc degeneration through TRPA1 methylation to inhibit the COX2/YAP axis" was retracted in 2024. Reasons: results that could not be reproduced; plagiarized images; overlap with other authors' work; signs of a paper mill.

### Methylation-specific PCR (MSP)

Genomic DNA was extracted from tissues and cells using a genomic DNA purification kit (Qiagen, Hilden, Germany). Bisulfite modification of DNA was performed by using the Intergen CpGenome DNA modification kit (Intergen, NY, USA) according to the instructions provided. DNA was evaluated by electrophoresis in a 3% Tris-borate-EDTA agarose gel and the gel imaging system to analyze the PCR products. TRPA1 methylation specific primers were designed through the Methprimer online program website (http://www.urogene.org/cgi-bin/methprimer/methprimer.cgi), M (F: 5'-TTGTAGTTGTAGGATAGCGGGAC-3', R: 5'-TTCTAAAAAAAATTCTCAAACCCG-3'), U (F: 5'-GTTGTAGTTGTAGGATAGTGGGATG-3', R: 5'-ACTTCTAAAAAAAATTCTCAAACCCA-3').

### Dual luciferase reporter gene assay

The promoter sequence of TRPA1 was retrieved from the National Center for Biotechnology Information (NCBI) database (http://www.ncbi.nlm.nih.gov/gene) (-2000 bp to 50 bp) and cloned to the PGL3-control vector to form PGL3-TRPA1-wild type (TRPA1-WT) plasmid. The sequence with a mutated binding site of DNMT3B and TRPA1 was synthesized to construct the PGL3-TRPA1-mutant plasmid (TRPA1-MUT). NP cells in the logarithmic growth phase were inoculated into a 6-well plate. The NP cells were co-treated with control + oe-NC, aza (aza: DNMT3B inhibitor) + oe-NC, control + oe-DNMT3B, aza + oe-DNMT3B, and TRPA1-WT or TRPA1-MUT after 24 hours of inoculation. After 48 hours, the dual luciferase assay kit (RG005, Beyotime Biotechnology Co., Shanghai, China) was used for the detection of luciferase activity.

### Western blot

After treatments, intervertebral disc tissues and NP cells were washed with cold PBS, lysed with cooled RIPA lysis solution plus 1 mmol/L PMSF, and centrifugated. The total protein content extracted from tissues and cells was separated by 10% sodium dodecyl sulfate polyacrylamide gel electrophoresis and transferred onto a polyvinylidene fluoride membrane; the protein concentration was determined by a protein determination kit (Bio-Rad, Richmond, CA, USA). Next, the membrane was immersed in TBST (25 mmol/L Tris, pH 7.5, 150 mmol/L NaCl and 0.1% Tween 20) containing 5% bovine serum albumin (BSA) for 1 hour. The membrane was incubated overnight at 4° C with primary rabbit antibodies against DNMT3B (ab239893, 1:1000, Abcam, Cambridge, UK), TRPA1 (ab58844, 1:500, Abcam, Cambridge, UK), COX2 (ab15191, 1:1000, Abcam, Cambridge, UK), YAP (ab205270, 1:1000, Abcam, Cambridge, UK), aggrecan (ab186414, 1:1000, Abcam, Cambridge, UK), collagen II (ab34712, 1:1500, Abcam, Cambridge, UK), MMP3 (ab52915, 1:2000, Abcam, Cambridge, UK), MMP9 (ab38898, 1:1500, Abcam, Cambridge, UK), Bcl2 (ab182858, 1:1500, Abcam, Cambridge, UK), caspase-3 (ab13847, 1:1500, Abcam, Cambridge, UK), Bax (ab32503, 1:1500, Abcam, Cambridge, UK), and mouse anti-GAPDH (ab205719, 1:1000, Abcam, Cambridge, UK). The membrane was then washed 3 times (5 minutes each time) by TBST, and incubated with horseradish peroxidase-labeled secondary antibodies goat anti-rabbit IgG (ab205718, 1:20000, Abcam, Cambridge, UK) and goat anti-mouse IgG (ab150117, 1:20000, Abcam, Cambridge, UK) for 1 hour. Finally, the blots were developed with enhanced chemiluminescence (Thermo Fisher Scientific, MA, USA), imaged by a Chemi-Scope mini-imaging system (Clinx Science Instruments Co., Ltd., Shanghai, China), and semi-quantified using ImageJ software (National Institutes of Health, Bethesda, MD, USA).

The article "DNMT3B decreases extracellular matrix degradation and alleviates intervertebral disc degeneration through TRPA1 methylation to inhibit the COX2/YAP axis" was retracted in 2024. Reasons: results that could not be reproduced; plagiarized images; overlap with other authors' work; signs of a paper mill.

### Reverse transcription quantitative polymerase chain reaction (RT-qPCR)

Intervertebral disc tissues and NP cells were incubated with Trizol Reagent (15596026, Invitrogen, Car, USA), and centrifuged at 4° C. The supernatant was centrifuged with chloroform to obtain total RNA. PrimeScript^TM^ One Step RT-PCR Kit (Takara, Shiga, Japan) was used for the reverse transcription of mRNA, with the reaction conditions set at 37° C for 15 minutes and 85° C for 5 seconds. RNA were subjected to RT-PCR reaction in a real-time qPCR instrument (ABI7500, ABI, Foster City, CA, USA) with the reaction system formed with SYBR Premix EX Taq kit (RR420A, Takara, Shiga, Japan). The relative expression was calculated by using 2^-ΔΔCt^ method with GAPDH as the internal reference gene. The primer sequences for RT-qPCR are listed in Table 1. The experiment was repeated three times.

**Table 1:** Primer sequences for RT-qPCR.

**Gene**	**Sequences**
DNMT3B	F: 5′-ACAACCATTGACTTTGCCGC -3′
	R: 5′-CGTTCTCGGCTCTCCTCATC -3′
TRPA1	F: 5′-CTGTGAAGCGCTGAATGTAATG-3′
	R: 5′-GCTCCTTGGCTGAGAAGAAA-3′
COX2	F: 5′-ATTCTTTGCCCAGCACTTCACT-3′
	R: 5′-CCTCTCCACCGATGACCTGATA-3′
YAP	F: 5′-ACCATAAGAACAAGACCACATCC-3′
	R: 5′-TTCAATCGCAGCCTCTCCTT-3′
Bax	F: 5′-TGTTACAGGGTTTCATCCAG-3′
	R: 5′-ATCCTCTGCAGCTCCATATT-3′
Bcl2	F: 5′-GATTGTGGCCTTCTTTGAGT-3′
	R: 5′-ATAGTTCCACAAAGGCATCC-3′
Caspase-3	F: 5′-GAAAGCCGAAACTCTTCATCA-3′
	R: 5′-ATAGTAACCGGGTGCGGTAT-3′
collagen II	F: 5′-CTTTCCTCCGTCTACTGTCCA-3′
	R: 5′-GCCCTCATCTCCACATCATT-3′
aggrecan	F: 5′-GGGACCTGTGTGAGATCGAC -3′
	R: 5′-GGTCGGGAAAGTGGCGATAA -3′
MMP3	F: 5′-GGACCAGGGATTAATGGAGATG-3′
	R: 5′-TGAGCAGCAACCAGGAATAG-3′
MMP9	F: 5′-AGCCGGGAACGTATCTGGA-3′
	R: 5′-TGGAAACTCACACGCCAGAAG-3′
GAPDH	F: 5′-ATGCCATCACTGCCACTCA-3′
	R: 5′-CCTGCTTCACCACCTTCTTG-3′

Note: F: forward; R: reverse.

The article "DNMT3B decreases extracellular matrix degradation and alleviates intervertebral disc degeneration through TRPA1 methylation to inhibit the COX2/YAP axis" was retracted in 2024. Reasons: results that could not be reproduced; plagiarized images; overlap with other authors' work; signs of a paper mill.

### Statistical analysis

All measurement data were processed using the SPSS 21.0 statistical software (SPSS, Chicago, IL, USA) and expressed as the mean ± standard deviation. Data between the two groups were analyzed by an independent sample *t*-test. Data between multiple groups were analyzed by one-way analysis of variance (ANOVA). Data between groups at different time points were analyzed by repeated measurements of ANOVA with Tukey's post-hoc test. *p* < 0.05 refers to a statistically significant difference.
